The article "Spinal Tuina Improves Cognitive Impairment in Cerebral Palsy Rats through Inhibiting Pyroptosis Induced by NLRP3 and Caspase-1" was published in 2021. Journal: Evid Based Complement Alternat Med.

# Spinal Tuina Improves Cognitive Impairment in Cerebral Palsy Rats through Inhibiting Pyroptosis Induced by NLRP3 and Caspase-1

**DOI:** 10.1155/2021/1028909

**Published:** 2021-10-14

**Authors:** Feng Niu, Cuiting Wang, Hequan Zhong, Ningna Ren, Xiaokun Wang, Bing Li

**Affiliations:** ^1^Department of Rehabilitation, Jinshan Hospital, Fudan University, Shanghai 201508, China; ^2^Research Center for Clinical Medicine, Jinshan Hospital Affiliated to Fudan University, Shanghai 201508, China; ^3^College of Acupuncture-Massage and Rehabilitation, Yunnan University of Traditional Chinese Medicine, Kunming 650500, China

## Abstract

Cerebral palsy (CP) is a severe cerebral disease with high mortality and morbidity, which leads to great challenges for the suffering children and their families. Hence, the need for the efficacious and safe treatments is urgent. As a physical therapy arising from traditional Chinese medicine (TCM), Tuina has shown multiple effects on various diseases, including cerebral palsy. Nevertheless, the detailed mechanisms of Tuina on CP remain unknown, which impedes its further clinical application. Herein, we explored the effects of Tuina on CP and its potential mechanisms. Thirty Sprague Dawley (SD) male rats were randomly divided into sham, model, and Tuina groups (model + Tuina). CP rat model was established by hypoxia-ischemia via permanent occlusion of left common carotid artery and hypoxia for 2.5 hours caused by anaerobic environment, which was subsequently followed by onset of Tuina treatment from postnatal day 7 (P7) to P49. After completion of Tuina treatment, the behavioral tests showed that Tuina treatment not only improved the retarded body weight and impaired motor balance function, but also ameliorated weakened learning and memory function of CP rats. Moreover, immunohistochemistry and western blot also revealed a reduced expression of NLRP3 inflammasome and corresponding pyroptosis-related molecules induced by NLRP3 in CP rats after Tuina treatment. Therefore, our study indicated that Tuina treatment may improve impaired neurocognitive function of CP rats, which was possibly realised via inhibiting NLRP3-induced pyroptosis.

## 1. Introduction

Cerebral palsy (CP), the leading cause of life-long disability in children [1], affects approximately 1 in 500 neonates with an estimated prevalence of 17 million people worldwide [2–4]. CP heavily burdens the families and society [5]. Among the various risk factors, perinatal hypoxic-ischemic encephalopathy (HIE) is an important etiological factor in neonatal CP [6]; therefore, a rat model of HIE is considered a relatively ideal CP model. On the one hand, although updated medications and physical and surgical methods have been administered and applied to CP patients, positive improvements have not been confirmed [7–9]. Therefore, it is essential to explore more efficacious therapies for CP.

The article "Spinal Tuina Improves Cognitive Impairment in Cerebral Palsy Rats through Inhibiting Pyroptosis Induced by NLRP3 and Caspase-1" was published in 2021. Journal: Evid Based Complement Alternat Med.

As a physical therapy derived from traditional Chinese medicine (TCM), Tuina has shown multiple effects on a diverse set of diseases, including CP—although the effects of Tuina in CP remain controversial. Previous studies have indicated that Tuina may be used to improve the cognitive and motor functions and self-care abilities of children with CP [10–13]. Nevertheless, the precise mechanism of Tuina to treat CP is still unclear, which limits its clinical application. Additionally, pyroptosis (a proinflammatory form of programmed cell death characterized by inflammasome formation, caspase-1 activation, and cytokine-mediated inflammation [14]) has been proven to be involved in a variety of diseases [15–17]. Multiple studies have revealed the participation of pyroptosis in central nervous system (CNS) diseases, such as ischemic insult and chronic neuroinflammation [17, 18]. NOD-like receptors (NLRs) are a large family of intracellular receptors, among which NLRP3 has been widely explored. A previous study indicated that inhibition of NLRP3 may attenuate neonatal HI-induced brain injury in rats [19]. Among the pyroptosis pathways, activation of the NLRP3 inflammasome plays a central role and eventually mediates subsequent caspase-1 activation, cytokine secretion, and cell death [20].

Therefore, the current study proves that Tuina may enhance the cognitive functions of cerebral palsy rats and further explore whether this effect is related to the inhibition of NLRP3-induced pyroptosis.

## 2. Materials and Methods

### 2.1. Animals and Grouping

Sprague Dawley (SD) rat male pups, three days after birth (P3), were purchased from Shanghai Jihui Experimental Animal Breeding Co., Ltd. (production license number: SCXK (Shanghai) 2017-0012). Thirty pups were randomly divided into the following groups: sham, model, and Tuina (model + Tuina group) (*n* = 10 for each group). All pups were fed by their mothers during the lactation period and housed in a controlled temperature (22 ± 1°C) and humidity (50 ± 10%) environment on a 12-hour light-dark cycle with freely available food and water throughout the study after the lactation period. The animal experiments were conducted according to the experimental animal welfare ethics and animal experiment safety regulations of Fudan University and were reviewed and approved by the Animal Ethics Committee of the Shanghai Public Health Clinical Center. The day of birth was regarded as postnatal day 0 (P0), and all pups were weighed every two days starting from P3.

The article "Spinal Tuina Improves Cognitive Impairment in Cerebral Palsy Rats through Inhibiting Pyroptosis Induced by NLRP3 and Caspase-1" was published in 2021. Journal: Evid Based Complement Alternat Med.

### 2.2. Neonatal Hypoxic-Ischemic Encephalopathy Animal Model

The HIE model was established as previously described in other studies. First, P7 rat pups in the model group and Tuina group were anaesthetized with isoflurane (3% induction and 1.5% maintenance). Then, the left common carotid artery (LCCA) was isolated, and electrocoagulation was performed to permanently block the blood flow in the LCCA. Subsequently, the skin incision was sutured, and these rat pups were placed at 37°C for recovery. After being awake from anesthesia for one hour, all of the rat pups were placed in an anaerobic (8% O_2_+ 92% N_2_, at 37°C) chamber for an additional 2.5 hours. The LCCAs of the pups in the sham group was exposed without any further manipulations.

## 3. Methods of Spinal Tuina

The specific performance of Tuina treatment is as follows. First, before the onset of Tuina treatment, each rat pup was placed on the left palm of the performer to adapt to the environment for 1 min. Then, the threaded surface of the thumb or middle finger was used to softly press and rub the middle of the spine of each rat, which is named the governor vessel in traditional Chinese medicine (TCM).Third, the same manipulation was performed on both sides of the spine along the bladder meridian. Finally, the heads and limbs of the rats were rubbed gently to cover the acupoints Baihui, Yintang, Shenting, Sishencong, Quchi, Waiguan, Hegu, Yanglingquan, Zusanli, Sanyinjiao, and Taichong. This Tuina treatment was performed once a day from P7 to P49 and lasted for approximately 20 min each time. No interventions were administered to the rats in the non-Tuina group.

### 3.1. Balance Beam Test

The balance beam experiment was used to measure the balance ability, muscle strength, and movement coordination of the rats. In this experiment, the rats were placed at one end of a beam (100 cm long, 2 cm wide, and 50 cm above the floor) and allowed to pass along the beam to the other end, which was located in a dark box. Training was conducted once a day from P40 to P42 to familiarize the rats with the beam. On the test day (P43), the time required to reach the dark box at the other end of the beam and the number of slips of the hindlimb paws were recorded. Prior to each trial, the rats were acclimatized to the experimental environment for 30 min. The beam and the dark box were cleaned with ethanol after each trial.

### 3.2. Light-Dark Box Test (LDB Test)

The light-dark box was composed of a box (45 cm × 27 cm × 27 cm) with two equally sized light and dark compartments interconnected by a tunnel (7.5 cm × 7.5 cm). On P44, the rats were brought to the testing room for 30 min of acclimatization and allowed to explore the device in the light box for 5 min before the trial. After the rats entered the dark box, the interconnecting tunnel was closed, and subsequently, an electrical stimulation of 0.5 mA was given that lasted for 2 sec. On P45, the rats were placed in the light box again, and the interconnecting tunnel was opened at the same time. The latency required for the rats to enter the dark box, the number of times the rats entered the dark box, and the duration the rats spent in each compartment were recorded over a period of 5 min. The box was cleaned with ethanol after each trial.

The article "Spinal Tuina Improves Cognitive Impairment in Cerebral Palsy Rats through Inhibiting Pyroptosis Induced by NLRP3 and Caspase-1" was published in 2021. Journal: Evid Based Complement Alternat Med.

### 3.3. Morris Water Maze Test

The Morris water maze (MWM) test was adopted to examine spatial learning and memory performance as previously described [21]. The MWM equipment consisted of a columnar pool 160 cm in diameter and 50 cm high and a circular transparent platform with a diameter of 10 cm, which was placed 1 cm below the water's surface in the target quadrant. The water was opaque by using an edible pigment and controlled at a relatively stable temperature (25 ± 1°C). During the training period from P46 to P49, the rats were trained to find the platform within 60 sec by the hints set around the pool or under the guidance of the experimenter if the rats could not find the platform. The rats were allowed to stay on the platform for 30 sec. Each rat was trained four times a day, with an interval of 30 min between each training session. On the test day (P50), the platform was removed from the pool, and then, the rats were placed on the opposite side of the platform at the midpoint of the quadrant wall. The time required for the rats to enter the platform location for the first time and the time spent in the target quadrant afterwards were recorded.

### 3.4. Immunohistochemistry

Staining procedures and protocols for immunohistochemistry (IHC) were performed as follows. First, the rats were sacrificed on P50 and perfused with 4% paraformaldehyde from the left ventricle for brain fixation. Subsequently, ethanol and xylene were used for gradient dehydration and hyalinization before embedding the brain in paraffin for sectioning. After being deparaffinized in xylene, the sections were rehydrated with ethanol, followed by high-pressure antigen retrieval performed in a 0.1 M sodium citrate solution. Subsequently, the naturally cooled sections were incubated with a 3% H2O2 solution for 10 min at room temperature and then blocked with 5% bovine serum in PBS at room temperature for one hour. Next, a rabbit anti-rat NLRP3 primary antibody (1 : 300, Abcam) was added, followed by overnight incubation at 4°C. Then, a goat anti-rabbit secondary antibody (1 : 200) was added after the sections were rinsed with PBS three times, and again, the sections were incubated at room temperature for one hour the next day. Ultimately, NLRP3 was visualized with DAB.

The article "Spinal Tuina Improves Cognitive Impairment in Cerebral Palsy Rats through Inhibiting Pyroptosis Induced by NLRP3 and Caspase-1" was published in 2021. Journal: Evid Based Complement Alternat Med.

### 3.5. Western Blotting

The expression levels of caspase-1, cleaved caspase-1, IL-1*β*, IL-18, and GSDMD were measured by western blot. The hippocampi of the rats were homogenized with ice-cold protein lysis solution and subsequently centrifuged at 12000 g and 4°C for 20 min to obtain the supernatant. A BCA protein quantitative detection kit was used to determine the protein concentration, and then, the protein samples were separated by electrophoresis on SDS-polyacrylamide gels and transferred to PVDF membranes. After being blocked with fat-free milk for one hour, the membranes were incubated overnight at 4°C with primary antibodies against NLRP3 (1 : 1000, Abcam), caspase-1 (1 : 1000, Affinity), cleaved caspase-1 (1 : 1000, Affinity), IL-1*β* (1 : 1000, Affinity), IL-18 (1 : 1000, Affinity), GSDMD (1 : 1000, Abcam), and GAPDH (1 : 3000, Affinity). Subsequently, secondary antibodies were added, and the membranes were again incubated at room temperature for one hour. ECL chemiluminescence reagent was used to visualize the protein bands. The relative densities of the protein bands were analyzed using ImageJ.

### 3.6. Statistical Analysis

All data are expressed as the mean ± standard deviation (SD), and SPSS 22.0 software was used for statistical analysis. The differences between the three groups were analyzed by one-way analysis of variance (ANOVA), while Tukey's test was used for comparisons between two groups. *p* < 0.05 was considered statistically significant.

## 4. Results

### 4.1. Tuina Treatment Improves the Increase in Body Weight

The weight changes of the pups in each group reflect their general growth and development. As shown in Figure 1, over the period of P3 to P5, there was no difference in the change in body weight among the three groups, whereas a significant decrease in weight changes was detected over the period of P7 to P15 (model group vs. sham group; Tuina group vs. sham group; *p* < 0.05). Moreover, the Tuina group displayed a significant increase in weight change compared with the model group over the period of P31 to P49.

### 4.2. Tuina Treatment Improves the Motor Performance of CP Rats

Motor performance was assessed by the balance beam test. As shown in Figure 2, the time spent by the rats crossing the beam in the model group was greater than that in the sham group (Figure 2(a); *p* < 0.05), which indicated motor deficits in CP rats. The rats in the Tuina group spent less time passing along the beam than those in the model group, whereas no significant difference was detected between the Tuina group and the Sham group. Similarly, the rats subjected to HI (i.e., the model group) showed more slips of the hindlimbs than the sham group of rats, and the number of hindlimb slips was significantly alleviated after Tuina treatment (Figure 2(b); *p* < 0.05).

The article "Spinal Tuina Improves Cognitive Impairment in Cerebral Palsy Rats through Inhibiting Pyroptosis Induced by NLRP3 and Caspase-1" was published in 2021. Journal: Evid Based Complement Alternat Med.

### 4.3. Tuina Treatment Ameliorates the Learning and Memory Functions of CP Rats

Spatial learning and memory functions and fear memory were appraised by the MWM test and LDB test, respectively. In the LDB test, we found that the number of rats in the model group entering the dark box was significantly greater than that of the rats in the sham group. Moreover, the rats in the Tuina group displayed fewer entries into the dark box than those in the model group (Figures 3(a)–3(d)), which suggested that long-term Tuina treatment may improve the learning and memory performance of CP rats. In addition, the latency time of the rats entering the dark box in the model and Tuina groups was longer than that in the sham group, whereas no significant difference was found between the model group and Tuina group (Figure 3(e)). In the MWM test, the CP rats (i.e., the rats in the model and Tuina groups) spent more time finding the platform than those in the sham group, whereas the rats in the Tuina group spent significantly less time finding the platform compared with the rats in the model group. Additionally, we found that CP spent a lower percentage of time in the target quadrant than those in the sham group (Figures 4(a)–4(d)), whereas the rats in the Tuina group displayed a higher percentage of time spent in the target quadrant than the model group (Figure 4(e)). All these data indicated that the learning and memory functions of CP rats were damaged and Tuina treatment partly reversed these learning and memory deficits.

### 4.4. Tuina Treatment Reduced the Expression of NLRP3 in the Hippocampi of CP Rats

Immunohistochemistry and western blotting were used to observe the location and expression of the NLRP3 inflammasome in the hippocampus. The immunohistochemistry results revealed that NLRP3 was mainly expressed in the cytoplasm (Figures 5(a)–5(c)), and the expression of NLRP3 was significantly higher in the model group than in the sham group and Tuina group, whereas no significant difference was found between the sham group and Tuina group (Figures 5(d) and 5(e)).

### 4.5. Tuina Treatment Influences the Expression of Pyroptosis-Related Molecules in the Hippocampi of CP Rats

Pyroptosis is a form of programmed cell death that shares some common features of both apoptosis and necrosis. Our findings indicated that the expression of some pyroptosis-related molecules changed after HIE modeling and Tuina treatment. The expression of caspase-1 was insignificantly different among the three groups, whereas the expression of cleaved caspase-1, IL-1*β*, IL-18, and GSDMD was higher in the model and Tuina groups than in the sham group (*p* < 0.05). In addition, the expression of these molecules was lower in the Tuina group than the model group (Figures 6(a) and 6(b)). These results indicated that, after the activation of the pyroptosis pathway in CP, Tuina treatment may decrease the expression of pyroptosis-related molecules to provide a neuroprotective function.

The article "Spinal Tuina Improves Cognitive Impairment in Cerebral Palsy Rats through Inhibiting Pyroptosis Induced by NLRP3 and Caspase-1" was published in 2021. Journal: Evid Based Complement Alternat Med.

## 5. Discussion

It is widely accepted that cerebral palsy (CP) not only manifests as a disorder of posture and movements but also involves many other impairments, including cognitive, linguistic, communicative, and sensory-perceptual disturbances [22], which exert detrimental influences on the psychological well-being and quality of life of children and heavily burden the families and society. To date, there are still very few effective treatments for CP, which stresses the significance of exploring safe and efficacious alternative therapies. Tuina, originating from traditional Chinese medicine, is a nondrug and noninvasive therapy. Tuina manipulations have been performed along specific channels (meridians) and on confirmed acupuncture points on the body surface of patients for the purpose of alleviating symptoms of diseases [23]. Some clinical trials have reported that Tuina is beneficial for motor function improvement, intellectual development, and improvement of self-care abilities and the daily life of children with CP [10, 24, 25]. Moreover, animal experiments have shown that Tuina improved the motor balance and cognitive functions of HIE rats, the underlying mechanism of which was associated with the regulation of inflammation and genome-wide DNA hydroxymethylation levels [13, 26]. However, these studies are far from adequate in terms of clarifying the mechanism of the therapeutic effects of Tuina. Thus, a multitude of studies are needed to explore the underlying mechanisms of Tuina on cerebral palsy and support the clinical application of Tuina.

In the present study, we clearly demonstrated that Tuina treatment improved the long-term cognitive functions of CP rats by inhibiting NLRP3-induced pyroptosis in the hippocampus. Our results showed that the cognitive function of CP rats was apparently improved by Tuina treatment. By measuring changes in the body weights of the rats, we discovered that the changes in the body weights of CP rats were significantly increased after Tuina administration, which suggested a beneficial effect of Tuina on the growth and development of CP rats. Moreover, cognitive development, including motor coordination and memory, was also appraised by a series of animal behavioral tests. As shown by the balance beam test, the rats in the Tuina group displayed significant decreases in the cross time and number of hindlimb slips compared with the rats in the model group, which signified that Tuina treatment improved the motor coordination of CP rats. Additionally, as indicated by the results of the LDB test, the Tuina group entered the dark box fewer times over the experimental period compared with the model group, which suggested that Tuina enhanced the memory of CP rats after electrical stimulation. Therefore, the rats in the Tuina group showed a reduced number of entries into the dark box, as the dark box was naturally more attractive to the rats that entered less frequently. The Morris water maze (MWM) test is a representative method to assess the learning and memory of animals [27]. As shown by the results of the MWM test, the Tuina group spent less time finding the platform and stayed longer in the target quadrant than the model group, which also demonstrated that Tuina improved the memory of CP rats.

The article "Spinal Tuina Improves Cognitive Impairment in Cerebral Palsy Rats through Inhibiting Pyroptosis Induced by NLRP3 and Caspase-1" was published in 2021. Journal: Evid Based Complement Alternat Med.

NLRP3 inflammasome activation and pyroptosis have been described in neonatal hypoxic-ischemic encephalopathy [28–31]. When danger signals (such as ischemia and hypoxia) appear, NLRP3, an intracellular sensor, is able to recognize these signals and forms and activates the NLRP3 inflammasome [32]. Assembly of the NLRP3 inflammasome regulates activation of the proteolytic enzyme caspase-1, which subsequently leads to caspase 1-dependent release of the proinflammatory cytokines IL-1*β* and IL-18 and gasdermin D-mediated pyroptosis [33]. Pyroptosis is a subtype of regulated necrosis characterized by the formation of plasma membrane pores, cell swelling, rapid plasma membrane rupture, and release of proinflammatory intracellular contents and cytokines [34]. Activation of NLRP3/caspase-1/IL-1*β* signaling has been confirmed to occur within 4 h of HI brain injury in neonatal rats [29]. It was previously discovered that the expression of the key molecules in the pyroptosis pathway in HIE patients increases, and their levels are tightly correlated with the severity of HIE. Thus, a pyroptosis inhibitor was applied to rats with HIE, and its ability to alleviate injury severity was confirmed [30]. It was also demonstrated that the level of the HSP90*α*/HSP90AA1 peptide in the cerebrospinal fluid (CSF) of neonates with hypoxic-ischemic brain damage (HIBD) was reduced by peptidome analysis, and this peptide was involved in the NOD-LIKE receptor (NLR) signaling pathway [28]. Briefly, NLRP3-activated apoptosis plays a critical role in the pathophysiology of CP induced by HI and leads to brain damage [30]. Some previous studies have confirmed that pyroptosis inhibition had positive impacts on the prognosis of HIE. In one study, an IRE1*α* inhibitor was proven to protect HIE rats by inactivating the NLRP1/caspase-1 pathway, and the NLRP1 activator CRISPR, which was used to activate NLRP1, offsets the protective effects of an IRE1*α* inhibitor [35]. In another study, it was shown that TIGAR played a protective role in neonatal HIBD by inhibiting microglial pyroptosis. In addition, the brain atrophy and infarct size of TRPV1 KO mice after HI were decreased, which was found to be closely related to suppressing the activation of astrocytes and releasing astrocyte-derived IL-1*β*, mainly via JAK2-STAT3 signaling and activation of the NLRP3 inflammasome [36]. There was also a study on the effects of TCM formulae on pyroptosis in which Buyang Huanwu decoction improved neurological dysfunction and inhibited neuronal pyroptosis in the hippocampal CA1 region following MCAO/R [37]. Additionally, it has been reported that acupuncture may attenuate cognitive defects in an Alzheimer's disease (AD) mouse model by inhibiting NLRP1 inflammasome-mediated pyroptosis [38], which is indirectly in line with our findings because both acupuncture and Tuina share the similar therapy mindset of stimulating meridians and collaterals along the body surface. Consistent with these studies, we showed that the expression levels of NLRP3, cleaved caspase-1, IL-1*β*, IL-18, and GSDMD in the hippocampi of SD rats significantly increased after the induction of ischemia and hypoxia. Pyroptosis of neuronal cells in the hippocampus leads to learning and memory disorders. Notably, Tuina may inhibit NLRP3-mediated pyroptosis in CP rats and, therefore, improve cognitive function. However, in the present study, we explored the possible mechanism of Tuina in cerebral palsy through the canonical pyroptosis pathway, although it is unknown whether other pathways, such as the noncanonical pyroptosis pathway, also play a role. Given the complex inflammatory reactions during the pathological process of cerebral palsy, our research is far from sufficient to establish a comprehensive understanding of Tuina in cerebral palsy.

The article "Spinal Tuina Improves Cognitive Impairment in Cerebral Palsy Rats through Inhibiting Pyroptosis Induced by NLRP3 and Caspase-1" was published in 2021. Journal: Evid Based Complement Alternat Med.

Furthermore, the current study was based only on animal experiments, while, for clinical treatment, more clinical research is certainly required. In summary, more exhaustive signaling pathways and the incorporation of the clinical efficacy of Tuina will be the main focuses in future work, which will shed light on the molecular mechanism and give momentum to the application of Tuina in the treatment of cerebral palsy.

## 6. Conclusion

Our study demonstrated that Tuina treatment significantly attenuated cognitive impairment in a rat model of cerebral palsy, which may be mediated by inhibiting NLRP3-mediated pyroptosis in the hippocampus. Therefore, it is worthwhile to conduct a further preclinical investigation on the therapeutic effects of Tuina in cerebral palsy.

## Figures and Tables

**Figure 1:** Tuina treatment improved body weight increase. The average weights of the rat pups (*n* = 10) were measured from P3 to P49, and hypoxia ischemia intervention was performed on P7. The body weight increase significantly dropped after HIE modeling and was partly ameliorated by Tuina treatment (both *p* < 0.05). Data are presented as the means ± SD; ^*∗*^*p* < 0.05 compared with the sham group; ^#^*p* < 0.05 compared with the model group.

**Figure 2:** Tuina treatment improved the motor performance of CP rats. (a) Time required for the rats to cross the beam (*n* = 10). (b) Number of slips of the hindlimbs of the rats. Based on the results of Figures 2(a) and 2(b), the Tuina group displayed better motor performance than the model group (*p* < 0.05). Data are presented as the means ± SD; ^*∗*^*p* < 0.05 compared with the sham group; ^#^*p* < 0.05 compared with the model group.

**Figure 3:** Tuina treatment ameliorated fear learning and memory functions of in rats. (a–c) The movement tracks of the rats in the three groups (*n* = 10). (d) The number of times the rats entered the dark box. (e) The latency time required for the rats to enter the dark box for the first time. These data indicated better fear learning and memory performance in Tuina group. Data are presented as the means ± SD; ^*∗*^*p* < 0.05 compared with the sham group; ^#^*p* < 0.05 compared with the model group.

**Figure 4:** Tuina treatment improved the spatial learning and memory functions of CP rats. (a–c) The movement tracks of the rats in all three groups (*n* = 10). (d) The latency time required for the rats to find the platform. (e) The percent time spent by the rats in the target quadrant after removal of the platform. The Tuina group displayed better learning and memory functions than the model group (*p* < 0.05). Data are presented as the means ± SD; ^*∗*^*p* < 0.05 compared with the sham group; ^#^*p* < 0.05 compared with the model group.

**Figure 5:** Tuina treatment reduced the expression of NLRP3 in the hippocampi of HIE rats. (a–c) NLRP3 was mainly expressed in the cytoplasm. (d) Western blot analysis of NLRP3. (e) Quantification of the expression of NLRP3 in the three groups. The expression of NLRP3 was reduced in the Tuina group compared with the model group (*p* < 0.05). Data are presented as the means ± SD; ^*∗*^*p* < 0.05 compared with the sham group; ^#^*p* < 0.05 compared with the model group.

The article "Spinal Tuina Improves Cognitive Impairment in Cerebral Palsy Rats through Inhibiting Pyroptosis Induced by NLRP3 and Caspase-1" was published in 2021. Journal: Evid Based Complement Alternat Med.

**Figure 6:** Tuina treatment influenced the expression of pyroptosis-related molecules in the hippocampi of HIE rats. (a) Western blot analysis of caspase-1, cleaved caspase-1, IL-1*β*, IL-18, and GSDMD expression six weeks after HIE. (b) Quantitative analyses of these pyroptosis-related molecules. Pyroptosis-related molecules were partly downregulated after Tuina treatment. Data are presented as the means ± SD; ^*∗*^*p* < 0.05 compared with the sham group; ^#^*p* < 0.05 compared with the model group.

## Data Availability

The data used to support the findings of this study are available within the article.
